This article has been retracted.

# Development and Teaching Application of Interactive Virtual Algorithm Animation of C Language Program

**DOI:** 10.1155/2022/7082914

**Published:** 2022-07-30

**Authors:** Lei Wan, Yongli Cao, Lili Shi, Ying An

**Affiliations:** Department of Animation, Qingdao Huanghai University, Shandong 266400, China

## Abstract

In today's world, almost every domain has certain and mandatory requirements to understand at least one of the programming languages which is defined as a way of interaction with a computer to resolve real world problems or more specifically for the implementation of algorithms. Language programming is a course with strong theory and practice. In view of the fact that C language beginners in colleges and universities generally report that it is difficult to learn well due to various reasons. Therefore, in this paper, we have discussed the development and teaching of interactive virtual animation of C language programs. The proposed approach relies on a typical recursive algorithm case to analyze the teaching strategy of virtual algorithm animation brought into the classroom, the application in the algorithm teaching of C language and the teaching strategy in improving students' understanding of abstract knowledge using computer C language program interactive virtual animation development and implementation of the teaching system is the research content. According to the basic flow of the interactive virtual algorithm of the C language program, a reasonable system structure design is carried out.

## 1. Introduction

In the twenty-first century, with the rapid development of computer multimedia technology, network technology and other information technologies and the implementation of the “information superhighway” cross-century project, today's information age has put forward new requirements for education. A programming language is a collection of rules for converting texts, or graphical programme components in the case of visual programming languages, into machine code. A programming language is a type of computer language that is used to implement algorithms in computer programming. Instructions for computers make up the majority of programming languages. Instead of using general programming languages, some programmable machines use a set of specific instructions. Nowadays, exploring new teaching and learning methods supported by information technology and cultivating new talents have become an important task for schools to adapt to the development of the times. The essence of information-based education is that it has an unprecedented and distinct service nature, which serves learning and learners. In view of this, Shanwei Vocational and Technical College proposes that higher vocational C language programming courses should carry out teaching reforms in terms of teaching concepts, educational theories, teaching methods and means, and teaching evaluation, focusing on cultivating students' autonomous learning ability, cognitive ability, collaboration ability, lifelong learning ability, and innovation ability, forming a good emotional attitude and values, etc., so as to promote the comprehensive and harmonious development of students.

Usually, information collected or fetched by human beings have various ways or simply, we can say it has numerous resources through which it can be extracted such as experimental psychologist Treicher. It has confirmed through a large number of experiments that approximately 83% of the information collected by human beings is collected through vision, 11% from hearing through ears. This mean through these two resources we are able to get a total of 94% of the overall needed information. Apart from it, another 3.5% of the information is obtained through another sense that is smell whereas 1.5% and 1% from touch and taste senses, respectively. In this way, the amount of information obtained through the stimulation of multiple senses is much stronger than simply listening to the teacher's lectures. Information and knowledge are closely related, and more knowledge can be acquired by acquiring a large amount of information.

In this paper, we study how to apply visual animation teaching strategies in the teaching of C language such that it enables students to explore, discover, understand, master, and use teaching content in the “virtual reality”, so as to achieve the purpose of cultivating students' creative quality and ability in a subtle way, is of great significance.

This article will be in J. Under the guidance of Sweuer's cognitive load theory, starting from the cognitive psychology of students, this paper discusses the application of game introduction teaching strategies in promoting the visualization of algorithmic teaching in C language.

The rest of the article is organized as given below.

In subsequent section, various definitions of the related terms are provided along with proper explanation where it is needed. Second, the application of game introduction teaching strategies is described and their importance in resolving the problem at hand is described. Results are presented in section 3, which is followed by the comprehensive and summarized form known as conclusion.

### 1.1. Definition of Related Concepts

An algorithm is a method, process, or idea taken to solve a problem. Likewise, an algorithm is defined as a way or step or path of solving particular problems which are written in the form of instruction or steps. It is the soul of the program, the program design depends on the algorithm, and the algorithm exists independently of the program. As long as you have mastered algorithm design, you can implement this algorithm in any computer language you have learned. The quality of the algorithm directly determines the running time of the entire program and the accuracy of the running result. It is important to note that algorithms is the main focus of teaching especially in situations of the programming courses or languages, but it is equally a tough and difficult to carry. Teaching strategy (instructional strategy) is a systematic decision-making activity by teachers in the process of teaching implementation according to the characteristics of teaching situations in order to achieve teaching goals. The teaching strategy of game introduction refers to the systematic decision-making activities in which teachers borrow or learn from the teaching of healthy and educational game software or courseware to stimulate students' desire for knowledge of course knowledge, and improve students' computer operation skills and skills through game operation.

### 1.2. The Application of Game Introduction Teaching Strategies

In the learning process of algorithms in C language, the algorithms to be learned are intertwined with the practical problems to be solved, and they interact with each other, creating a high level of intrinsic cognitive load in the students' minds. According to J. According to SweIIer's cognitive load theory, if the internal cognitive load is high (i.e., complex and difficult learning content), and the external cognitive load is also high, then the total cognitive load will exceed the total intellectual resources, and learning may fail. Excessive levels of cognitive load may arise directly from the instructional material presented to students, and instructional design that reduces extrinsic cognitive load can facilitate learning; content areas most likely to benefit from improved instructional design are those that need to deal with complex The field of information, and the algorithm learning of C language belongs to this field.

Therefore, if teachers pay more attention to teaching design, present teaching materials in a systematic and organized manner, and effectively display teaching resources in a visual form, through the interaction of vision and thinking, it should be able to reduce the cognitive load of learners and allow students to focus on for protestant learning content, ensure that as much working memory as possible is released for encoding the information to be learned, increasing learning outcomes. Moreover, through this, students can understand how to analyze and solve practical problems and cultivate students' correct thinking mode of programming. Different strategies can be adopted in the teaching of different contents. This paper will take a typical recursive algorithm as a case to analyze the application of teaching strategies in the algorithm teaching of C language.

The Tower of Hanoi problem is a classical mathematical problem that can only be solved by recursive methods. Here, we choose it as an example for further studying the recursive algorithm.

In teaching, strategies introduced by games to help with problem solving are used, allowing students to explore and discover learning. There are conflicts and differences between the initial state and the target state. In an attempt to solve a well-known problem, i.e., tower of Hanoi, the respective students have to select a precisely accurate choice among the different possibilities which are available. Additionally, these students are further pressurized by the restriction that their choice or selection must be precise and accurate as wrong choices are misleading. Thus, we can conclude that decision making and thinking are among the remarkable manifestation of students' subjective initiative especially in these scenarios. On the other hand, in the process of problem solving, it has gone through several processes from the preparation stage to the gestation stage, the sudden stage, the evaluation and correction stage, which is exactly the process of creative thinking. Creative thinking is a high-level form of human thinking. It is also the teaching goal.

## 2. Design Concept of the Virtual Algorithm

### 2.1. Algorithm Design Goals

On the basis of realizing the computer networking, which is primarily defined as how a group of electronic devices are connected to form an operational network especially for sharing of resources and data, of each learning link including the corresponding management functions, the automation degree of the system and the operating performance of the system are improved [1]. Thus, the system user identity is automatically identified. Moreover, random and subjective questions are automatically evaluated whereas online scores is automatically generated.

In order to ensure the security and confidentiality of the test questions in the test question bank, the system has designed the feature of automatic identification of user identities, so that different users have different permissions and can perform different operations [2].

In the specific environment of the computer room, in order to ensure that the test questions of the students and the neighboring candidates are different, to prevent cheating, and to ensure that the test questions have the same difficulty coefficient, in the process of automatic test composition, the characteristics of random questions are fully considered to ensure the fairness of the test sex.

The automatic evaluation of subjective questions in the system is mainly used in the programming part. The automatic evaluation of subjective questions is different from the automatic evaluation of subjective questions in some examination systems. The automatic evaluation of subjective questions is limited to the characteristics of the comparison program results [3]. In addition to comparing the results, the automatic evaluation of subjective questions in this system can further check and correct small errors in the program and can match keywords for programs that cannot run results. Scores that are closer to the results of manual evaluation, thereby reducing the workload of teachers' evaluation.

Teachers' burden to tally students' grades is substantially reduced by the feature of automated creation of online grades. The results of each portion of the applicants' exam questions are directly entered into the grade sheet after the automatic evaluation [4], and the class grade sheet is prepared for instructors and students to query.

The online examination system's security and dependability are critical to the system's ability to function regularly. The test is quite important. Incidents such as the leakage of test questions are never permitted in order to maintain the fairness of the exam [5]. As a result, other encryption safeguards must be incorporated in addition to employing the database's security mechanism to secure the exam questions stored on the server side. Identity verification, permission setting, and stopping unauthorized users from assaulting and stealing should all be included in the system [6].

### 2.2. Algorithm Development Tools

The server-side operating system platform selects Microsoft's Windows2003Server, and selects SQL Server2000 as the database management system to ensure the large capacity and high security of the database; the application program is programmed with the VB6.0 programming language as the development tool. Each client uses the Windows XP operating system.

When designing and developing an application system, no matter which structure is adopted, it depends on the network configuration, application requirements, function realization, and other factors of the system. The key technology to realize the online examination system is the use of database in the network environment [7, 8], so the problem comes down to the question of how to choose the architecture of the database system. Currently throughout the world, most of the examination system's structure consist of C/S and B/S structures which are equally important in their own way.

B/S structure: This structure is suitable for the development of the Internet. The biggest advantage is that the client does not need to install software, as long as there is IE to run, so it can be used in the actual network with a long distance, making the most of it. The biggest disadvantage is that the data security is low, the server requirements are high, and the data transmission speed is slow.

C/S structure: This structure is a traditional structure, the technology is very mature, it has a safe access mode, the network traffic is low, and the response speed is fast. The disadvantage is that the client program must be installed, and the maintenance is difficult and costly.

The structural design of this system is based on the hardware and software of the computer room, the situation of maintenance personnel and the requirements of the examination system itself. The computer room is equipped with a full-time technical teacher [9], and each machine has a recovery card. After the first installation and configuration, there is no need to repeat the settings for the subsequent exams, which makes up for the structural shortcomings. The operation object of the examination system is a large number of students, so it has high requirements for speed and security. In these two points, the B/S structure is far less than the C/S structure, so the C/S structure is considered comprehensively. The design can better meet the actual needs of the system.

According to the specific use environment, the system adopts the structure mode based on local area network as shown in Figure 1.

In this system, the complete system is further divided into two subsystems which are according to the user type (i) Teacher (administrator) and (ii) Examinee subsystems respectively. The teacher subsystem mainly completes system management, user management, examination management, test question management, test paper management, and score management; the candidate subsystem mainly implements online examinations. According to two different subsystems, the system is divided into several functional modules.

Before determining the functional modules of the system, we first analyze the needs of the system. Because the test is oriented to a specific object, the online test is carried out. Since the test environment is generally a computer room, and the distance between each test taker is very close, in order to ensure the safety of the test paper and prevent the test taker from cheating [10], the test paper obtained by each test taker The type and size of the questions should be the same and the difficulty of the questions should be the same, but the content of the questions is not the same.

The online test is based on the network environment, and the test papers that can meet the above requirements should be generated dynamically after randomly extracting test questions from the server's database. In addition, the system should also control the test time [11]. When the time is up, the test will be required to be handed in or forced to stop the test. After the test taker chooses the answer and submits it, the computer will automatically judge the paper and get the score statistics.

Teachers must be able to insert, add, remove, and alter test questions at any time and from any location in these systems, particularly through the examination system's administration terminal and with the permission of the administrators. He or she also has the authority to interfere in the knowledge points and question size, as well as to review the exam results [12].

In addition to realizing the above functions, the online examination system should also have a friendly and concise interface, high security, and strong stability.

## 3. Implementation of Interactive Algorithm Technology

### 3.1. Implementation of Automatic Volume Grouping

The user enters the specific requirements for the test paper to be generated, and the computer converts these requirements into quantitative parameters such as difficulty, knowledge points, and scores of each category or topic in the test paper [13], and then extracts the test questions according to a certain algorithm. The test questions are compared with the assessment conditions, and if the assessment fails, the questions will be re-selected. After the test questions are selected, test papers are generated by arranging test questions and assigning scores as shown in Figure 2.

In order to make the system automatically form a test with moderate difficulty and a wide coverage of knowledge points, the system is designed based on the difficulty coefficient. Important points of the coverage topic selection method:

1. Initialize: in this step, a temporary test question table is created or generated that is initially empty, a temporary test question bank table and import all the questions of this type of knowledge points that have not been extracted in this subject.
2. Take the group roll parameters: Take out the parameters of a certain question type in the group volume strategy table
3. Analysis and calculation: Determine the number of questions and other parameters of the required various difficulty coefficient test questions according to the extracted test set parameters.
4. Take the test questions: Combined with the random number selection and the parameters to be introduced below, the qualified test questions will be taken from the temporary test question bank. The ones that have not been drawn will be given priority.

By analyzing various question types, it is found that the comprehensive test questions are programming questions because the parameters of the test are relatively clear [14], the number of questions is small, and the extraction is relatively easy. Therefore, in the actual test composition, the test questions of the programming questions are matched first and then match the simple type of questions. First, the knowledge points are sorted in the descending order of their scores, and the question types under the knowledge points are also arranged in descending order of their scores. If there are no questions matching the control parameters in the question bank, the control parameters will be relaxed [15]. The average difficulty coefficient of the test paper is guaranteed by the difficulty coefficient of each knowledge point. After all the questions of the knowledge point are drawn, if the error of the difficulty coefficient is within the allowable range, proceed to the next knowledge point; otherwise, use the corresponding strategy to optimize and adjust the difficulty coefficient of the knowledge point.

### 3.2. Automatic Random Topic Selection Based on an Interactive Algorithm

The automatic grouping of papers not only ensures that all papers have the same level of difficulty but also ensures that the questions in the papers cannot be repeated. Therefore, in addition to meeting the parameters set in the test set record, it is also required that the test papers produced each time cannot contain the same questions. In order to ensure this principle, the function RandA is designed using Vb. The function of the function is to randomly select *m* (*m* ≤ 11) different numbers from *n* different numbers (that is, to select *m* different test questions from the questions). The core code is as follows:

- function RandA(*n* as integer, *m* as integer, b())
- *j* = *O*
- count = *O*//Counter initialization
- If *m* > *n* then msgbox'‘project error!!”
- for *i* = Oton—l step 1
- a(*i*) = 0//Initialize the array a and set all numbers to the unselected state
- next i
- while(count ≤ *m*)//Select *m* number
- *j* = n *∗* RndO//Generate a belly, a random number between n-1. while(A(*j*) = 1)//If *j* has been selected, point *j* to the next number
- *j*=(*i*+1)mod n
- wend
- a0) = *l*//until an unselected *j* is found, set its selected flag to 1
- count = count + 1//Counter increments by 1
- wend
- count = *O*
- for *i* = Oton-l step 1
- if a(*i*) = 1 then
- *b*(count) = 1//Store the selected number in the array *b*
- count = coqu *t* + *l*
- endif
- next *i*
- end function

The objective function of this problem is as follows:

(1) $$\begin{array}{c} T=\min\left(\max\left(T_{ij}+p_{ij}\right)\right),\\ \min T_{ij},\\ V=\min\overset{n}{\underset{j=1}{\sum }}v_{j},\\ T_{ci\left(j+1\right)}\geq T_{cij}+P_{cij},\\ T_{xy}\geq \max\left(T_{ij}+P_{ij}\right). \end{array}$$

During automatic test composition, we first save the test question numbers of the 11 test questions that meet the test composition record in the array A with *n* elements, and then call the function R and A to get the array B with *m* elements, and the values of the elements in B are all Less than or equal to *n*, that is, the value of the element in B is t subscript of the element in A. According to the value of the element in B, the corresponding subscript element in A is obtained, and the value of the element is the number of the selected test item. Then, we read the detailed content of the test item from the test item information table according to the test item number, store it in the test paper list, and number it in sequence.

For example: get *n* = 5 from the query; and *A* = {”12”, “107”, “219”, “112”, “314”}; and get *m* = 3 from the volume record; call the function RandA to get *B*=(1, 3, 4); then, according to the values in A(1), A(3), A(4), the question numbers are read from the question information table as “12”, “219”, “112” The detailed content of the test questions, i.e., these three test questions, are selected test questions.

The application is based on the difficulty scale. Whether the test paper automatically composed of knowledge point coverage and automatic random number-based topic selection algorithm can truly reflect the teaching level of teachers and students' mastery of knowledge and skills requires us to evaluate the quality of test papers [16]. The main test indicators for measuring the test papers are: difficulty and coverage. We set the number of questions in the test paper to be sampled as *n*, based on the M-point system, and the full score for each question is *A*_j_(*j* = 1,2,3, ..., n); the capacity of the random check is N, and the sample value is *X*_i_(*i* = *l*, 2, 3, ..., N) is the number of test papers for random inspection; The actual score of each question in the N test papers is X_ij_(*i* = *l*, 2, 3, ..., N; *j* = 1, 2, 3, ..., n); then, the sample value is as follows:

(2) $$\begin{array}{c} X_{i}=\sum_{j=1}^{M}X_{ij},\;\left(i=1,2,3,\ldots ,N;j=1,2,3,\ldots ,n\right). \end{array}$$

The average of the jth question is ${\bar{X}}_{j}=\left(1/N\right)\sum_{i=1}^{N}X_{ij}$, The variance of the jth problem is $S_{j}=\left(1/N\right)\sum_{i=1}^{N}{\left(X_{ij}-\bar{X_{j}}\right)}^{2}$.

The computer itself is a very large runtime system for applications written in machine instructions. The instructions in the application program are executed on the computer by a physical central processing unit (cpu, Central Processing Unit), and the specific process of executing the program on the computer is managed by the operating system. Therefore, this type of runtime system is composed of computer hardware itself and software. That is to say, a virtual machine of abstraction is added between the computer and the compiler. This virtual machine provides a common interface to the compiler on any platform. The compiler only needs to face the virtual machine, generate code that the virtual machine can understand, and then the interpreter converts the virtual machine code into machine code for a specific system. Implement. The code that this virtual machine can understand is called bytecode, and it is not oriented to any specific processor, only to the target virtual machine. The interpreter for each platform is different, but the virtual machine implemented is the same. After the source program is compiled by the compiler, it becomes bytecode, and the bytecode is executed by the virtual machine. The virtual machine sends each bytecode to be executed to the interpreter [17], and the interpreter translates it into a machine code on a specific machine. Then, we run it on a specific machine. A virtual machine is an abstract computer that has an instruction set and uses different storage areas like a real computer. It is responsible for executing instructions, but also managing data, memory, and registers [18].

Finally, a virtual machine is a computer system that has been virtualized or emulated. Virtual machines are built on computer architectures and provide actual computer functions. Specialized hardware, software, or a combination of both may be used in their implementations. The virtual machine system is a collection of standards rather than a simple software implementation. Any programme that wishes to function on a virtual machine must rigorously adhere to these criteria, and only in this way can applications be smoothly migrated from one platform to another. The Sun Java Virtual Machine, which debuted in the 1990s, is a notable example of this. We can witness the large software system developed by the Java standard in numerous commercial application software today [19].

## 4. Virtual Algorithm Animation Implementation Process

The students were also thinking actively during the repeated game process, which laid a good foundation for the smooth programming of the subsequent programs. Next, the teacher and the students conducted an algorithm analysis together. Most of the students said that although the moving process is very complicated and cumbersome, the regularity is very strong: to use the recursive calling technology to solve this moving process, first find a recursive calling model. To get a simple solution to the Tower of Hanoi problem, the focus should be to move the large plate at the bottom of the A-bar, not the small plate at the top.

The general case of *n* disks instead of 64 disks is considered. To move n-1 discs on the A rod to the C rod, think of it like this:

**Step 1 .**

With the help of the *c* rod, first try to move n-1 disks from the A rod to the B rod, as shown by the arrow ① in Figure 3.

**Step 2 .**

Move the remaining nth disk in the *A* rod to the *C* rod, as shown by the arrow ② in Figure 3.

**Step 3 .**

Move the n-1 disks on the *B* block to the *c* rod with the help of the A rod, as shown by the arrow ③ in Figure 3.

As shown in Figure 3, most of the students expressed their understanding. The first and third steps are to move n-1 disks from one pole to another. The method is the same, but the pole names are different. Now, the first and third steps are general. It can be expressed as: move n-1 disks on the “one” rod to the “two” rod (with the help of the “three” rod), move n-1 disks on the “no” rod to the “three” rod (with the help of the “three” rod) “one” lever). In the first and third steps, one, two, and three have different correspondences with *A*, *B*, and *C*. In the first step, the corresponding relationship is one-*A*, coffee-*B*, and three-*C*. In the third step, the corresponding relationship is one-*B*, two-*C*, and three-*A*.

Two functions are used to realize the above operation: we use the hanoi function to realize the operation of moving n-1 disks from one rod to another rod, which is a recursive process, hanoi (*n*, one, two, three) means “put *n* The plate is moved from the one rod to the three rod (with the help of the tw0 rod)”. We use the move function to implement the operation of moving a disk from one rod to another.

Write the program as follows:

  void hanoi (int *n*, char one, char two, char three)
  {if(*n* = = 1) printf(”%c- ->%c\n”, one, three);.
  else{
  hanoi(n- 1, one, three, two);
  printf(”%c ->%c \n”, one, three);
  hanoi(n- 1, two, one, three);
  }
  main
 
*n*()
  int *m*;
  scanf(”%d”, and m);
  hamoi(m,‘A',‘B',‘C');
  }

Compared with traditional teaching methods, the teaching strategies introduced by games can stimulate students' interest in learning and promote students' image thinking. Creativity, students constantly develop decision-making thinking through continuous thinking in repeated games. Combined with appropriate dynamic interactive prompts on the screen, they can test the accuracy of their thinking in real time, and constantly judge their own ideas. In the process of problem solving, students went through various stages of creative thinking, gave full play to their initiative and creativity, deepened their understanding of algorithms, and achieved very effective learning results.

## 5. Conclusion and Future Work

In this paper, we study how to apply visual animation teaching strategies in the teaching of C language such that it enables students to explore, discover, understand, master, and use teaching content in the “virtual reality”, so as to achieve the purpose of cultivating students' creative quality and ability in a subtle way, is of great significance. Initially, through a large number of tests, the interactive virtual algorithm animation has created a new, autonomous learning, and free exploration learning space for C language programming algorithm teaching, which is one of the effective ways to solve the difficulty of algorithm teaching. It gives ideal results and participates in vision and hearing to grasp key and difficult points faster, which is not only conducive to the assistance of teachers in explaining algorithms in class but also suitable for students' self-learning operations.

In future, its extended application is not only suitable for the algorithm teaching of C programs but also for the teaching of algorithms in other programming languages such as VB, VF, *C* + +  and other similar courses.

## Figures and Tables

**Figure 1:** Flowchart of the hybrid teaching optimization algorithm.

**Figure 2:** Volume flow chart.

**Figure 3:** Tower of Hanoi game.

## Data Availability

The datasets used and analyzed during the current study are available from the corresponding author upon reasonable request.
